The article "Capturing potential impact of challenge-based gamification on gamified quizzing in the classroom" was retracted in 2026. Reason: lack of ethics approval or compliance.

# Capturing potential impact of challenge-based gamification on gamified quizzing in the classroom^☆^

**DOI:** 10.1016/j.heliyon.2021.e08637

**Published:** 2021-12-20

**Authors:** Punyawee Anunpattana, Mohd Nor Akmal Khalid, Hiroyuki Iida, Wilawan Inchamnan

**Affiliations:** a School of Information Science, Japan Advanced Institute of Science and Technology, 1-1 Asahidai, Nomi, 923-1211 Ishikawa, Japan; b Research Center for Entertainment Science, Japan Advanced Institute of Science and Technology, 1-1 Asahidai, Nomi, 923-1211 Ishikawa, Japan; c College of Creative Design and Entertainment, Dhurakij Bundit University, Bangkok, Thailand

**Keywords:** Gamification, Physics in mind, Quizzing, Engagement, Time pressure, Challenge adjustment

## Abstract

Challenges in education have continuously been addressed by integrating gamification, but a gap remains for game design principles that support user engagement. This paper outlines results obtained from integrating challenge-based gamification into an elementary school classroom to examine the emergence of student engagement and learning-related behavior. The approach was applied to logical puzzle quizzes where different gamification adjustments were captured and examined using physics' analogy (called the motion in mind concept). The structural experiment, with a mixed methods design, was designed around the notion of time pressure and the difficulty of gamifying the quizzing experience. This model was constructed to validate and expand the quantitative findings (motion in mind model) by including qualitative explorations (thematic analysis). The results revealed the potential synthesis of motion in mind and flow theory, and its relationships to engagement and learning were identified as a new conceptual scheme.

## 1 Introduction

Education is currently facing global challenges, and studies are continuously being conducted to improve its quality by means of developing technologies and integrating effective methods for improving learning outcomes and engagement in both the short and long term (Sanchez et al., 2020; Dichev and Dicheva, 2017). Gamification plays a role as a motivator that facilitates and incorporates game elements into a nongame context, and is generally applied in the education aspect.

According to the gamification literature, gamification has been used mostly in education to understand the relationships and provide empirical support in this field, which has been applied in several studies (Hitchens and Tulloch, 2018; Bigdeli and Kaufman, 2017; Surendeleg et al., 2014; Simões et al., 2013; Nicholson, 2013; Deterding et al., 2011). Gamified education platforms have been employed to study the effect of gamified learning and engagement, since it can be easily shaped and configured in a variety of subjects and introduce game elements into classrooms without any effort. Using a gamified platform as a formative assessment platform encourages students to engage in the learning environment (Zainuddin et al., 2020; Wang and Tahir, 2020); it enables them to develop their performance to accomplish the tasks or activities. Likewise, a gamified platform can expose the merits and shortcomings in the game design level and contribute to fostering curiosity and assessing informative learning process (Laine and Lindberg, 2020; Zainuddin et al., 2020; Deterding et al., 2011).

In this study, we examined relevant articles, and found over 100 based on keywords such as gamification, education, and classroom. Previous field studies took advantage of the impacts of gamification: most studies adopted statistical inferences and psychological methods. One of the most influential works in this field was inspired by the flow concept (Nakamura and Csikszentmihalyi, 2014), where the understanding of the challenge in games that drives a sense of flow and engagement was met with the improvement of the player's skill level. The theoretical foundations of gamification research mainly rely on self-determination theory, which argues that intrinsic motivation can emerge to lad the individual to engage in activities that satisfy three basic psychological needs: autonomy, competence, and relatedness (Deci and Ryan, 2012). However, the existing studies did not provide comprehensive guidance for educational gamification design, which is still required for consolidating other theoretical approaches and domains. Most game designs provide the ability to adjust the level of difficulty according to the player, and individuals may tackle increasingly tricky challenges with higher levels of skills (Legaki et al., 2020; Hamari et al., 2016; Chang et al., 2018). Once reaching the flow, it often implies that the player intrinsically experiences a sense of enjoyment and satisfaction (Nakamura and Csikszentmihalyi, 2014). However, practical guidelines to use this as a motivator in gamified platforms are still lacking.

In this study, a gamified quizzing platform, Kahoot!, was employed to enhance engagement and learning performance based on the concept of motion in mind (Iida and Khalid, 2020). This paper presents three types of challenge adjustment: time pressure, difficulty, and adaptation of patterns. Various quizzing parameters were considered, such as the number of questions, time required for each question, and degree of difficulty. Hence, the goal was to empirically determine formative support of challenge-based gamification in an education context. Additionally, the impact of challenge-based gamification based on the motion in mind concept was identified, and the engagement and curiosity levels of quizzing as a gamified platform were evaluated.

Based on these premises, we intended to capture the impact by applying different variations of challenge-based gamification, including time pressure, difficulty levels, and gamified adaptation. This research addresses the following research questions:

1. How can engagement and learning performance enhance a gamified quizzing platform when considering the motion in mind concept to empirically measure the learner's experience?
2. How does challenge adjustment induce the expected engagement and learning performance? Are there any significant aspects of these three proposed experiments?
3. What are the impacts and perceptions of the student of the associations in gamified learning platforms using challenge-based gamification?

## 2 Background

### 2.1 Defining gamification

Gamification introduces a method of incorporating game mechanics and applying them to the nongame context to elicit user engagement and satisfaction. Several definitions have been widely defined in many domains, generally considered as applying game-based thinking through intrinsic and extrinsic motivation to enhance the overall performance of and engage the users (Laine and Lindberg, 2020; Surendeleg et al., 2014; Dichev and Dicheva, 2017; Kéri, 2019; Nicholson, 2013; Deterding et al., 2011; Klock et al., 2020). In the context of the current study, game-based learning is contrasted to the concept of gamification, which focuses on behavioral changes and is specifically developed to achieve a specific game outcome (Kéri, 2019; Kristen DiCerbo, 2016).

Fundamentally, the idea of gamification mostly comprises three main game design elements: the dynamics, mechanics, and components of the game (Table 1) (Deterding et al., 2011). These elements develop user engagement and encourage user enjoyment and curiosity. For example, ranking can increase competitiveness amongst users (Bicen and Kocakoyun, 2018; Zainuddin et al., 2020). As another example, a loyalty program can be more effective when a point or tier system is appropriately incorporated (Xin et al., 2018). To apply gamification, understanding user demands and driving factors is crucial, and those factors should be merged and combed relative to the game mechanics (Inchamnan and Anunpattana, 2019; Anunpattana et al., 2019). However, it is impossible to use all gamified elements within a single game. Therefore, careful consideration of the goal of gamification is important (Hursen and Bas, 2019).

**Table 1:** Game design elements (Deterding et al., 2011).

Dynamics	Mechanics	Components
Constraints	Challenges	Achievements
Emotions	Chances	Avatars
Narratives	Competition	Badges
Progression	Cooperation	Collections
Relationship	Feedback	Unlockable Content
	Resources	Leaderboards
	Rewards	Dashboard
	Turns	Levels/Tiers
	Win-Lose status	Points/Scores
	Exchange	Virtual Goods

### 2.2 Related work on gamification design

Many gamification designs have been constructed for various nongame contexts, such as education, in attempts to reconcile game elements toward particular objectives (Hitchens and Tulloch, 2018; Laine and Lindberg, 2020; Surendeleg et al., 2014); for health purposes, to incentivize the users (Chen and Pu, 2014; Cotton and Patel, 2019); marketing (Hamari et al., 2018; Mitchell et al., 2020); business (Deterding et al., 2011; Thavamuni et al., 2019); and sports (Dale, 2014). Furthermore, gamification concepts are incorporated into most applications, such as educational games (Bigdeli and Kaufman, 2017; Annetta, 2010; Hamari et al., 2016), hotel loyalty programs (Xin et al., 2018), frequent flier programs (Zuo et al., 2019), and resource conservation campaigns (Hamari et al., 2018).

The potential of gamification has been used to improve education, where its implementation must demonstrate an improvement in incentive, as a short-term consequence, and learning outcome, as a long-term consequence (Sanchez et al., 2020; Dichev and Dicheva, 2017). Many design principles have been proposed and categorized into several directions to identify an effective method to support the applicability of gamification (Laine and Lindberg, 2020; Klock et al., 2020). Researchers found that the challenge design principle can more easily engage diverse players than other principles (Legaki et al., 2020). Another study (Denisova and Cairns, 2015) reported that the game's challenge had positive effects on learning and engagement. The game's challenge is a reasonably strong motivator that produces different motivational results that depend on the context of use. Some studies applied gamification design through different strategies relative to the game-based learning processes only as a process or a tool to encourage motivation (Kéri, 2019). Additionally, game-based learning and an educational game were proposed as an activity (Laine and Lindberg, 2020). For instance, Minecraft has typically been considered a classroom tool that focuses solely on transferring the student's knowledge, which can be called game-based learning (Weitze, 2016): this gamification design idea had an integrated motivator that contributes to activity engagement.

One study showed how gamification can help children with dyslexia transition from primary to secondary school using an intervention technique (Gooch et al., 2016). Several researchers (Decker an Lawley, 2013; Hamari et al., 2014) explained that while there is the potential for gamification to promote short forms of motivation, the effect of gamification is dependent upon the application context (Seaborn and Fels, 2015). Additionally, an example of popular gamified educational systems (e.g., the Khan Academy) supports the benefits of increasing student motivation or generating learning-related outcomes in the early stages of education (Antin and Churchill, 2011); some extant research examined gamification targeted to increasing the amount of effort applied in activities related to these goals (Brewer et al., 2013; Domínguez et al., 2013). Aa qualitative study of an intervention on a gamified platform to learn algebra was conducted (Sætre, 2013). Finally, some studies on the impact of motivational approaches used commonly accepted categories of strategies such as competition, simulation, tangible rewards, or association (Hamari et al., 2014; Kankanhalli et al., 2012; Orji et al., 2017).

Given the previous research in this area, we found a research gap regarding the validation of gamification techniques' impacts on learner motivation and engagement using a mathematical model. As such, we applied a structural experiment approach to understand the implications of the popular gamification platform Kahoot on student motivation in the context of gamifying classrooms. The findings encourage others to employ challenge-related mechanics approaches to understand how authentic, unpredictable, and diverse pedagogical practices influence classroom effectiveness and gamification interventions.

### 2.3 Game design principles

Game design principles (Laine and Lindberg, 2020) should be applied to achieve a sense of challenge and the possibility of connecting relevant factors to outline the interpretation of challenge-based game design. Firstly, activities should include challenges with different difficulty levels, beginning with tutorials and beginner-level challenges to appeal to different players' varying skill levels. Tasks or activities can drive the player to the edge of their abilities while avoiding challenges that are either too simplistic or too complex. This reflects the difficulty underlying the aims of challenge-based gamification design, consisting of the critical component of the user being in the flow state. A challenge appropriate for the students' skill level must be provided. Secondly, adequate time could be designated to emphasize the impact of using a challenge-based approach since sufficient time pressure is helpful for reflection in a specific learning scenario. Finally, the adaptation can lead to feelings of competence and curiosity, which result in subsequent motivation to engage in the gamified activity. Therefore, these principles can help users overcome and encourage the state of mind by adding variation and unpredictable challenges.

Quizzing is the best way to employ gamification, using one type of test and evaluation that aids teachers and educators to understand the knowledge acquisition (Susanto and Yosephine, 2019). Quizzing is defined as a low-stake test that can enhance learning performance and help students retain their motivation, and the quizzing benefits can be clarified by manipulating the quiz frequency and placement to show significant learning improvements and exam performance both before and after a lecture (McDaniel et al., 2011). Gamification in quizzing has been investigated to determine its relative effectiveness (Cheong et al., 2013), its effects and as enabler of children's interaction and learning performance (Wang et al., 2016; Zainuddin et al., 2020), its improvements of engagement (Zainuddin et al., 2020), and its impacts on short-term assignments (Sanchez et al., 2020). However, the gamification effects in long-term and classroom settings are unclear since it may encourage various behavioral changes. Therefore, gamification requires an effective design that is dynamic and customizable (Kéri, 2019; Sepulveda et al., 2019; Klock et al., 2020).

Although previous studies have addressed essential aspects regarding gamification design, a gap remains regarding the game design principles that support user engagement, specifically in classroom gamification. Thus, this gap must addressed to determine and verify game design characteristics and methods in practical education, which was the core focus of this study.

### 2.4 Challenge-based gamification and its applications

Most previous studies discovered that complex activities and challenging aspects can be used to more deeply engage students, thus supporting the theory behind the concept of flow (Nakamura and Csikszentmihalyi, 2014). Users engagement and concentration are significantly correlated with the activity's level of challenge. A challenge is a solicitation to engage in a complex but achievable task. Uncertain outcomes are challenging because of the user's responses, various goals, hidden information, and randomness (Wilson et al., 2009). In Kankanhalli et al. (2012), users were driven by challenges to complete predefined tasks that helped inexperienced users to learn how to progress. This usually involves competence related to the basic psychological needs defined by self-determination theory (Deci and Ryan, 2012). The goal of this gamified approach was to acquire abilities by conquering challenging tasks. When the challenge is appropriate for the player's ability level, the challenge is a factor motivating improvements in competence.

In general, there are several methods of establishing challenges in a single-player game. Firstly, the difficulty can be fixed, and the users enjoy the game, but no sign of either skill development or engagement is found (Bicen and Kocakoyun, 2018; Legaki et al., 2020; Wang and Tahir, 2020). Secondly, if the difficulty gradually increases as the player advances, engagement is encouraged and learning performance is improved due to diversity of change of challenging arrangements (Sepulveda et al., 2019; Klock et al., 2020). Finally, the difficulty is balanced using the computational intelligence method (Denisova and Cairns, 2015), where games automatically adjust the difficulty based on evaluating various players' actions during the game. With this technique, games are becoming interactive, through which the player can be engaged with the environment created from the game based on their skill level.

These challenge-based gamification merits were found, in a classroom setting, to transform the learning situation into an engaging experience that encourages independence and self-competence (i.e., Weitze (2016) partitions the game into many iterations). Other studies focused on the quality of the education and the evaluation of the learning perceptions (Simões et al., 2013; Annetta, 2010; Jaeger and Adair, 2017). As a finding, engagement and performance were associated with the student's ability perception.

Proposition 3 from the theory of gamified learning proposed by Landers (2014) states that “game characteristics influence changes in behavior”. This proposition has been extended to many contexts, and especially in the educational context, for instance, in a training program (Farcas and Szamosközi, 2014) and in an educational environment (Canhoto and Murphy, 2016) to support learning engagement and potential relevance. The process of changing game elements may encourage student behaviors throughout the activity, and it can reflect the impact of the occurrences of engagement and learning progress. To summarize, challenge-based gamification may encourage a student to complete more tasks with higher motivation, a higher sense of achievement, and a better sense of learning progress, in which those elements are scrutinized through the motion in mind concept and flow theory. Table 2 describes the role of gamification components and design elements in this experiment, along with their summarized purposes for this study.

**Table 2:** Integrated game design elements in the challenge-based gamified quizzing.

Design Elements	Description	Purpose
Timer	Numeric measure of player's performance (time used)	Indicator of time pressure
Points, Scores	Numeric measure of player's performance (answer corrected)	Indicator of explicit reward
Levels	Difficulty level of quizzing provides the sense of progression	Indicator of progression and difficulty

## 3 Game refinement theory and motion in mind

### 3.1 Gamified experience and game progress model

A general model of game refinement, based on a logistic model of game uncertainty, was proposed by Iida et al. (2004). From the players' viewpoint, the information regarding the game result is an increasing function of time *t* (i.e., the number of moves in board games). Here, the information on the game result is defined as the amount of solved uncertainty (or information obtained) x(t), as given by (1). The parameter *n* (where 1≤n∈N) is the number of possible options, x(0)=0, and x(T)=1.

(1) $$x^{\prime }(t)=\frac{n}{t}\;x(t)$$

where x(T) is the normalized amount of solved uncertainty. Note that 0≤t≤T, 0≤x(t)≤1. Equation (1) implies that the rate of increase of the solved information $x^{\prime }(t)$ is proportional to x(t) and inversely proportional to *t*. By solving (1), (2) is obtained. It is assumed that the solved information x(t) is twice derivable at t∈[0,T]. The second derivative of (2) indicates the accelerated velocity of the solved uncertainty along with the game progress, which is described by (3). The acceleration of velocity implies the difference in the rate of acquired information during game progression. Then, a measure of game refinement *GR* is obtained as the root square of the second derivative, described by (4):

(2) $$x(t)={\left(\frac{t}{T}\right)}^{n}$$

(3) $$x^{\prime \prime }(t)=\frac{n\;(n-1)}{T^{n}}\;t^{n-2}{|}_{t=T}\;=\frac{n\;(n-1)}{T^{2}}$$

(4) $$GR=\frac{\sqrt{n\;(n-1)}}{T}$$

Let *p* be the probability of selecting the best choice among *n* plausible options. As such, the definition of gamified experience is based on the notion of the risk frequency ratio or risk-taking probability, which is defined as $m=1-p=\frac{n-1}{n}$ (Iida and Khalid, 2020). Then, the gamified experience is achieved if and only if the risk occurs with parameter m≥0.5, which implies n≥2. Knowing that the parameter *n* in (4) is the number of plausible moves, for a game with branching factor *B* and length *D*, $n≃\sqrt{B}$ is approximated where the *GR* is given as (5):

(5) $$GR\approx \frac{\sqrt{B}}{D}$$

In this paper, the ratio of solving rate is given as *v* and the solved uncertainty of the game y(t) is an increasing function of time *t*, which can be described by (6). A player may feel informational acceleration, which is formulated analogically to the physics formulation of motion $y(t)=ut+\frac{1}{2}at^{2}$. Since *u* is the initial velocity at t=0, then (7) is obtained. The intersection can be calculated at t=D or t=T, where (8) is identified as the informational acceleration that describes the gamified experience and comfortable thrills under consideration.

(6) y(t)=vt

(7) $$y(t)=\frac{1}{2}at^{2}$$

(8) $$a=\frac{2v}{D}=\frac{2v}{T}$$

Sophisticated games possess an appropriate game length to solve uncertainty while gaining the necessary information to identify the winner (Iida and Khalid, 2020). This condition can be found at the cross-point area between (6) and (7), where $a=\frac{B}{D^{2}}$ is identified as the noble uncertainty zone (∈[0.07,0.08]) of the $GR=\sqrt{a}$, as previously found (Table 3). Then, interpretation in the education context can be inherently conducted. As such, p=v and *m* are defined as the learning rate (ability) and the rate of solving the question correctly (capability) and difficulty (challenge), respectively.

**Table 3:** Measures of game refinement of major board games (Sutiono et al., 2014).

Game	*B*	*D*	GR	*a*
Western Chess	35	80	0.074	0.00547
Chinese Chess	38	95	0.065	0.00423
Japanese Chess	80	115	0.078	0.00608
Mah Jong	10.36	49.36	0.078	0.00608
Go	250	208	0.076	0.00578

### 3.2 Motion in mind

In physics, the fundamental element was measuring the mass and velocity, enabling the derivation of force, momentum, and potential energy. Intuitively, Table 4 illustrates an analogical link that relates physics in mind notations and its in-game counterparts (Iida and Khalid, 2020). Based on such analogy, various motion in games can be determined, where the momentum, potential energy, and force were defined as (9), (10), and (11), respectively.

(9) $$\overset{\to }{p}=m\cdot v$$

(10) $$E_{p}=ma\cdot y(t)=ma\left(\frac{1}{2}at^{2}\right)=\frac{1}{2}ma^{2}t^{2}=2mv^{2}$$

(11) $$F=ma=(1-v)\cdot a\;\mathrm{and}\;a=\frac{B}{D^{2}}$$

**Table 4:** Analogical link between physics and game (adopted from Iida and Khalid (2020)).

Notation	Physics context	Game context
*y*	Displacement	Solved uncertainty
*t*	Time	Progress or length
*v*	Velocity	Solving rate
*M*	Mass	Solving hardness, *m*
*g*	Acceleration (gravity)	Acceleration, *a* (thrills)
*F*	Newtonian force	Force in mind (move ability)
$\overset{\to }{p}$	Momentum	Momentum (move intensity)
*U*	Potential energy	Potential energy, *E*_*p*_ (move potential)

Previous works (Agarwal et al., 2019) showed that $\overset{\to }{p}$ represents the player's growth rate determined by the different game depth and change over time. In this paper, $\overset{\to }{p}$ signifies the users' capability to play the game. In the game process, the game's energy reflects the amount of the movement potential (anticipation or curiosity) that the game may transfer to the player (Iida and Khalid, 2020). In a game context, the definition is based on the notion of movement potential, which attracts players like gravity. A certain amount of anticipation is required in a skill-based game so that challenge contributes to the expected risk (a larger *m*). This situation implies more chance to progress in the game (high $E_{p}$), and anticipation decreases if the player acquires sufficient information; thus, the player perceives it as motivation to move (i.e., results in a desirable outcome). The concept of motion in mind of the engagement zones, demonstrating winning engagements (*m* < 0.2), involves highly addictive public gambling games that possess high game motivational potential (peak $E_{p}$ is located at m=0.33) whereas playing engagement mostly involves competitive games possessing high mind motivational potential (peak $E_{q}$ is located at m=0.67), with beginner-accessible games located at the peak of the negative force $F_{2}$ (Khalid and Iida, 2021). Fig. 1 plots the reward quantity against the solving uncertainty *m*, which depicts the characteristics and relationship between objectivity and subjectivity over the value *m*.

**Figure 1:** The states plotted against the difficulty of solving uncertainty in a game (*m*).

### 3.3 Law of conservation, engagement, and challenge-based gamification

In this paper, the potential energy ($E_{p}$) is conserved over time and transforms into the momentum of the game's motion and momentum of the mind's motion, from which a new measurement of engagement is determined. Analogous to the law of conservation of energy in classical physics, $E_{p}$ is expected to be conserved, where the momentum of the game playing motions, while differing in level, contains both objective (in-game) and subjective (in-mind) recognition.

Potential energy ($E_{p}$) is transformed into the momentum of the game's motion ($\overset{\to }{p_{1}}$) and the momentum of the mind's motion ($\overset{\to }{p_{2}}$), i.e., $E_{p}=\overset{\to }{p_{1}}+\overset{\to }{p_{2}}$. Hence, it is expected that $\overset{\to }{p_{2}}$ is a reliable measurement of engagement. Applying (12) and (10), (13) is obtained. Then, the first derivative of (13) is solved, where $m=\frac{3\pm \sqrt{3}}{6}$ is obtained and represents high excitement ($m=\frac{3+\sqrt{3}}{6}$) and high expectancy ($m=\frac{3-\sqrt{3}}{6}$). Hence, $\overset{\to }{p_{2}}$ has two peaks in different directions where play engagement is maximized.

(12) $$\overset{\to }{p_{1}}(m)=m\cdot v$$

(13) $$\overset{\to }{p_{2}}(m)=E_{p}-{\overset{\to }{p}}_{1}=2m^{3}-3m^{2}+m$$

Considering the objective momentum $\overset{\to }{p_{1}}$ and subjective momentum $\overset{\to }{p_{2}}$, $v_{1}$ and $v_{2}$ are the win rate (or velocity) for the objective and the subjective motions, respectively, being functions of mass *m*, given by (14) and (15). Then, the acceleration of the subjective motion $a_{2}$ is given by (16). Based on the acceleration of the subjective motion $a_{2}$, the game's subjective force ($F_{2}$) can be determined, described by (17). As previously defined (Iida and Khalid, 2020), force in mind indicates the player's ability to move in the game or relative to the player's strength in general. Solving $F_{2}=8m-3$, $m=\frac{3}{8}≃0.38$ is obtained as the lowest point of $F_{2}$ (negative peak). Such a peak implies that the game pushes the player to acquire the necessary ability instead of requiring the player's ability to move the game ($F_{1}$), making it a suitable condition for a novice or for educational purposes. Fig. 2(a) illustrates various objective and subjective motions of a game over various difficulties (*m*).

(14) $$v_{1}(m)=1-m$$

(15) $$v_{2}(m)=2m^{2}-3m+1$$

(16) $$a_{2}(m)=4m-3$$

(17) $$F_{2}=m\cdot a_{2}=m\cdot (4m-3)$$

**Figure 2:** An illustration of (a) the analogy of various physics measures over various masses (*m*), and (b) extended game progress model based on solved uncertainty (*y*).

In this paper, the challenge-based gamification relative to the various analogies of motion and its conservation is considered by translating the quizzing activities into two types of quantities: game refinement (*GR*) and velocity (*v*). From an information science point of view, the quizzing activities are considered a linear amount of solved uncertainty. Adopting game refinement theory can be considered as gamifying the activity or the accelerated amount of solved uncertainty (i.e., Δ*v*). Incorporating challenge-based gamification imitates both Δ*v* and Δ*a*, which generates vibration or jerk (*j*) in the activity's progression. Jerk represents sudden changes in thrills and engagement experience relative to the retention of motivation (Iida, 2008; Iida and Khalid, 2020). This situation is illustrated in Fig. 2(b).

Researchers Hoffman and Nadelson (2010) defined the conscious awareness of motivation for a particular action as motivational engagement. The strength of this awareness affects a player's perceptions of their ability to control the game process and their chances of winning. According to the study, pregaming decisions (such as game genres and enthusiasm in the activity) and “opposing interference force towards positive objectives” (such as mastering the game and overcoming challenges) are crucial contextual engagement gaps between gaming and education domains.

When playing competitively and collaboratively, it was demonstrated that involvement was higher when more substantial social exchanges, dialogues, and mutual glances warranted more effort (or arousal) (Arellano et al., 2016). Additionally, autonomy has a significant impact on engagement due to its ability to alter difficulty levels and increase intrinsic motivation for learning, both of which are subject to change over time (Leiker et al., 2016).

Engagement is a critical emotive component that is strongly linked to motivation and flow, controlled partly by difficulty, competence, tension, and escapism. Depending on the intake of other emotive components in game-playing UX and behaviors, engagement and addiction could be considered two sides of the same coin: addiction is equated with the negative side of engagement, such as relapse, conflict, inadequacy, and withdrawal. However, as inferred in previous studies, distinguishing engagement and addiction typically produces inconsistent findings and involves many overlapping affective components. A game should be designed so that the difficulty suits players' skills: not too complicated or too simple. In other terms, this condition is associated with the sense of control, making the game-playing experience engaging. A rational gaming-related decision influenced by inadequacy may result in a suboptimal outcome (King et al., 2018). This phenomenon is related to the sense of focus that makes a game-playing experience more attractive to the players and conceivably makes them invest more time in the game, thus being more associated with player satisfaction, which varies with gaming situation.

In the context of motion in mind, Khalid and Iida (2021) stated that motivation is associated with the potential energy ($E_{p}$), which addresses the weight of the play's progress and the player's expectation. Control and focus were associated with the velocity (*v*) and momentum ($\overset{\to }{p}$), which represent the rate of an individual's progression and activity, respectively. Additionally, challenge-based gamification was input to investigate the progression and performance of individual students. This can be considered the necessary factor for analyzing transition gamification regarding the motion in mind concept. Therefore, a conceptual model linking motion in mind to such psychological attributes based on previous studies was constructed, as depicted in Fig. 3.

**Figure 3:** The conceptual model of engagement and addiction by Khalid and Iida (2021) with challenge-based gamification.

## 4 Methodology

We designed an experiment to perform a challenge-based gamified assessment quiz system via Kahoot! to analyze the behavioral outcomes. In the experiment, the time pressure factor was first exerted by adjusting the time for each question. Then, the difficulty was adjusted based on predefined settings. Finally, an adaptation of patterns that randomized difficulty distribution and subgoal distribution were conducted. The behavioral changes among the various settings of the quiz were observed.

### 4.1 Mixed methodology

Mixed-methods research was employed in this study: quantitative information (i.e., gamified quizzing) ghat was gathered in the first stage was subsequently supported by qualitative data (interviews) in the second stage. Both quantitative and qualitative research questions were investigated and validated by implementing a triangulation design: validating quantitative data model, where information is administrated both concurrently and separately without correlation. However, this method design was applied based on the dominant-less dominant design in which the priority of the quantitative method is more pronounced than the qualitative method. This model was used to validate and expand the quantitative findings by including a few qualitative explorations.

Quantitative study data were collected from the experimental process via the metrics mentioned in the assessment section (Section 4.6). Qualitative data were collected to determine the depth of view in engagement improvement and learning improvement in the gamified quizzing context, and interviews were randomly conducted among the participants, forming the independent and dependent variables, respectively. Neither type of data collection interfered with the other in the study and the data were analyzed separately. Finally, the data were associated in order to respond to the research inquiries. Fig. 4 displays the triangulation methodological process in this study (Venkatesh et al., 2013).

**Figure 4:** A triangulation mixed-methods design. We adopted this research design to support the three experiments conducted in this study. The first experiment involved applying the time pressure factor, followed by difficulty adjustment in the second one. Thirdly, an adaptation of patterns that randomized difficulty distribution and subgoal distribution was conducted for the third experiment. Finally, these experiments were supported by another layer of assessment procedures, as described in Section 4.4.

We chose to use this design in this study, firstly, to combine the different strengths as well as the nonoverlapping weaknesses of quantitative and qualitative methods (Welch and Patton, 1992) and to triangulate the methods in order to directly compare and resolve conflicts between qualitative and quantitative findings (Chu and Chang, 2017). Quantitative information was obtained to verify our hypothesis in the theoretical point of view, developed by qualitative information. Secondly, this design was used to obtain insight into the same relationships' views. A qualitative study was used to gain insights complementary to the findings from the quantitative data. Therefore, the mixed method is characterized as developmental and complementary.

### 4.2 Variables and participants

The independent variables were the challenge intervention adjustment: time pressure, the difficulty of quizzes, and gamified adaptation. The dependent variables were the correctness (amount of correct answers during the session) and achievement time (amount of time used during the session). These parameters were analyzed via motion in mind to quantify student engagement. As such, other dependent variable was student engagement in the quizzing.

A total of 120 Thai elementary school students (n=120) from five different classes participated in this study. The students were aged between 7 and 12 years and were asked to take the gamified quiz during class time. All participants (n=120) were assigned the same experiment of three challenge-based gamification in this research. They were voluntarily recruited with a declaration to find the participants whose qualifications matched the study, and their written consent from their guardians was obtained. In this study, we followed the principles that all participants must be informed and highlighted all the negative and positive aspects of the research during the consent process, including revealing the objectives and nature of the research to the participants (Parveen and Showkat, 2017; Davis and Waycott, 2015).

The first experiment applied the time pressure factor, followed by the difficulty adjustment in the second experiment. Then, an adaptation of patterns that randomized difficulty distribution and subgoal distribution was applied for the third experiment. Pre- and post-test experiments were set up by pre-evaluating the performance and engagement through the score and time used before gamified elements were excluded, and post-evaluation after implementing the gamified elements was included. Multiple-choice quizzes (generally four choices) were conducted on the participant's device in real-time (tablet or computer). This pre- and post-test allowed us to obtain the results of using such gamification. Such interventions caused a shift in motivation and engagement. As such, the experiment focused on changing the parameters and inputting new adaptations related to challenge-based gamification to determine its suitability, which would affect the engagement and achievement of the participants. Therefore, the experimental methods in this study were used to confirm the potential impact through gamification and to determine the fundamental optimal point of incorporating gamified elements such as a challenge.

This study provides a remedy by using the same number of questions *N*, amount of time per each *t*, and difficulty level in three different experiments. Ten random participants (n=10) were invited to be interviewed regarding their learning and perceived experiences of the gamified quizzing. Two participants were randomly assigned from five different classes to discover the diverse impacts amongst the five different classes to obtain various information. The interviewees had different demographics, such as age and baseline capabilities (education level of elementary students). Concerning the ethical issues of the study, a heavy disguise strategy (Bruckman, 2002; Spicker, 2011) was adopted since the quantitative data were collected directly from the user interactions with the quizzing platform through their dashboard and leaderboard. Additionally, any related information that could identify the participants personally in the interviews was excluded unless explicit consent was given when recounting the responses.

### 4.3 Gamified platform: Kahoot!

Kahoot! is a free educational tool that educators use in schools, work presentations, and home learning via quizzes and interactive media^1^ (Plump and LaRosa, 2017). Kahoot! users can add pictures or videos and select the total time the players have to answer each question (5 to 120 s). Each question is worth up to 1000 points, divided by four choices with their respective marks. Points are assigned for a correct answer based on the answering speed; the faster an answer is given, the higher the score (Wang and Tahir, 2020). The results are shown on the screen when all participants have finished all the questions. The number of correct and wrong answers and lists of players with the most points (leaderboard) was shown on the screen (Bicen and Kocakoyun, 2018). Therefore, time and difficulty level were the parameters considered in this gamified platform. The screenshot of platform interface is shown in Fig. 5.

**Figure 5:** A screenshot of the Kahoot! user interface.

In the current study, challenge-based gamification was employed to reflect and capture student engagement and learning impact with quizzes. The primary outcome in our proposed approach is dependent on the alteration of each game design element. Student participation in the gamified activity was expressed by a higher number of correct answers and time used in the three different alterations throughout the experiments.

### 4.4 Procedures

A one-group pretest–post-test design was set up using two segments for pre- and post-treatment using our proposed challenge-based gamification intervention. The participants in the nontreatment group conduct the premeasurement test without a timer, with simple questions and nongamified quiz. This premeasurement could be considered as traditional quizzing. Then, the participants participated in all three experiments, which were implemented as separate sessions for each class. All of the conditions were implemented with the same group of students (n=120) with various challenge-based gamification approaches, allowing for comparisons and capturing the effects of various game elements on student engagement and achievement. The experimental processes for quantitative data were situated as depicted in Fig. 6. The experiment was conducted three times with the same group of students to observe students' interaction and growth performance each time (Nand et al., 2019).

**Figure 6:** A one-group pretest–post-test design for the quantitative experimental study.

The first experiment started to capture the impact of engagement and motivation in the classroom, focusing on time pressure. By considering time pressure as a challenge, a balance should be struck between the degree of time pressure and the competence of participants to achieve the goal under that time pressure. The primary goal of this experiment was to investigate the impact of time pressure in gamified quizzing on player engagement and achievement. If these links were found to exist, the next goal was to identify the optimum solution between time pressures and motivation, flow, engagement, and performance (quiz completion time). In the experimental conditions, a timer was employed to simulate time pressure in the game. The experiment conditions were set up by setting the time for answering questions *t*, the total time for the whole session *T*, and the number of questions *N*. The results of all three trials were averaged, and data were collected based on the achievement rate (time used *AT*). This included recording the number of questions the participants correctly answered.

The second experiment was conducted to investigate the impact of changing the difficulty level of quizzes, focusing on the complexity and difficulty that reflect individual skills and performance. The experiment conditions involved setting the given time for answering questions *t*, the total time for the whole session *T* scheduling, and the number of questions *N*. Additionally, the set of questions was adjusted from easy to hard to investigate the impact of increasing the challenge level during quizzing. We averaged the results from all three trials, and data were collected based on the performance (correctness or correct answers *c*). However, the difficulty level was the same, but the questions were varied each time in order to avoid the rote memorization problem.

The third experiment addressed gamified adaptation, in which we altered the game mechanics to analyze the potential of game elements, which were included in this study as randomization and subgoal achievement. For the adaptation, we modified the game elements and the traditional quizzing mechanics to different styles. Notably, challenge-based gamification in quizzing based on the effects of gamification diminishing over time was observed to have a significant impact. Eventually, these two adaptations were inferred as the sense of progression and contingency.

First, we integrated these game elements for randomization since they had the most influence on making each session look different. The experimental conditions including the time given for answering questions *t*, the total time scheduled for the session *T*, and the number of questions *N* were sett up. Additionally, the set of questions was adjusted to be easy, medium, or hard to investigate the impact of increasing the difficulty of quizzing. Th results from the three trials were averaged, and data were collected based on the achieved performance (correctness or correct answers *c*). Unexpected events were caused by randomization in the first adaptation, which created uncertainty and challenge. This mechanic was critical for mirroring the simultaneous time pressure and difficulty adjustment. The difficulty level was random, and the questions were different each time in this part. Because of the characteristics of random-based activities, frustration is a critical issue to handle, as a learner who is too frustrated with the game will abandon it. The balance between skill and challenge should be considered. The main purpose of this adaptation is having the student master all inherent mechanics within the gamified adaptation.

The difficulty level would be ideal for addressing the subgoal, depending on the participant's skills. This mechanic in the second adaptation provided feedback regarding who chose a wrong answer and increased the level of difficulty experienced by students during the quiz. The learning principle of this game mechanic is that repetition helps with memory and feedback helps people learn from their performance. Once the first question is answered correctly, the user is able to answer all subsequent questions correctly. The main aim of this adaptation was to understand the quiz contents in order to acquire cognitive knowledge. The scoring algorithm was not applied in this part: only whether the answer was correct was provided. This method produced a high-risk challenge throughout the session that would help stimulate engagement and learning.

### 4.5 Data collection

Data were collected based on the achieved performance (correctness) and rate (time used) in the post-measurement stage. We observed the impact of the gamification approach on the motion in mind parameters, which can be interpreted differently from various different potential capabilities and engagement perspectives. The score and time obtained were calculated using the proposed progress model in the assessment section. Data were directly collected from the platform to avoid vulnerable and marginalized gaps, and the data were altered and were reported to the participants after each session.

In this study, the control variables were held constant using the experimental protocols for all participant sessions. For instance, the instructions and time spent on an experimental task were the same for all participants during gamified quizzing, since we were constructing a method of measuring and capturing the impact through occurrences of engagement and achievement. In each experiment, number of questions *N*, the amount of time per question *t*, the difficulty of questions, and the questions set for all participants were established to minimize the potential interference induced by different procedures and characteristics, which were all set via the gamified platform.

Qualitative data were collected to empirically support the analytical validity from the theoretical perspective, as shown in Fig. 7. We asked 6 questions to the 10 participants (n=10) to collect qualitative study data. Ten participants comprised the gamified treatment group: the interviews were set up for participants who were involved in all gamified conditions. In this study, semistructured interviews were used to specify the areas to be addressed and allow the interviewer or interviewee to following an idea or response in greater detail (Venkatesh et al., 2013). This interview format is flexible, allowing participants to explore or elaborate on vital information. Qualitative interview techniques are thought to provide a deeper grasp of social processes than simply quantitative methods. There were two alternatives provided for participants: a personal interview or an online interview. Personal interviews were face-to-face for those who were available to attend the interview on a particular day. Online interviews were conducted as live streaming video for those who were not available on that day using Zoom. Interview length varied according to the participant, and all sessions were available to be conducted in the Thai or English language depending on the participants. Interviews typically lasted 15–20 min for both in-person or online interviews, through which we obtained deeper information and ensured that the participants understood the questions. The interview process continued after the quantitative parts were finished, and the data were analyzed by focusing on the themes of challenge-based gamification impact, experiences, and relationship to motion in mind theory. Suggestions or other comments were collected if they were associated with positive or negative outcomes, leading to new research findings involving time pressure, difficulty, and gamified adaptations. We used these questions to complete this concept and bridge the gap between its commonalities and flow theory by focusing on key terms and all relating interview scripts, including engagement and learning impact, inductively. The questions asked were open-ended, objective, sensitive, and straightforward (see Appendix A).

**Figure 7:** A flowchart for our qualitative experimental study using interviews.

The questions began with what the participants experienced and took away from the methodological experiment, which the participants could quickly answer before proceeding to more complicated or subjective matters. This can put respondents at ease, gain their confidence and familiarity, and generate rich data to help with the interview progress. This procedure was also conducted and followed after the quantitative experiment. Before an interview, respondents were briefed about the study's objectives and assured of ethical norms such as anonymity and confidentiality. Various skills and approaches must be used to collect comprehensive and representative data throughout an interview to ensure the participants understand (Venkatesh et al., 2013). The moderator of the interview helps participants to clarify their ideas and asks if they have any additional remarks at the end of the interview. Reflecting on the comments of participants and making probing remarks were adopted to help students understand the process, ensuring the participants were not intimidated. The root questions were allowed to be altered depending on the participants' perception. It is a good idea to ask respondents for clarification if the answer is ambiguous. This typically leads to the discovery of new, unexpected knowledge. This is subject to ethical norms that researchers must uphold, including the principles of integrity, honesty, objectivity, and openness (Parveen and Showkat, 2017). These questions were constructed to consider the impact after applying gamified quizzing to subjectively capture both user engagement and learning impact. A theoretical discussion was employed to obtain in-depth information to obtain our findings in quantitative analysis.

Quantitative and qualitative data were merged to validate the results and draw meta-inferences, gaining additional insight or new interpretations. We assumed that challenge-based gamification could reinforce the positive feedback in the sense of behaviors and outcomes. Data were collected throughout the gamification process with different adaptations. As such, different adaptations could be compared and investigated. After collecting data, the analysis process began.

### 4.6 Quantitative analysis and assessment

The quantitative data analysis process was conducted based on the parameters of the motion in mind concept. This section provides our essential insights into the general model constructed in this study. Engagement level was assessed using the motion in mind concept, which required interpretations of various values to validate the context to be addressed in the discussion. Learning impact is not clearly defined. We graded the qualitative analysis and the behavioral changes observed therein to fill this gap. This measurement provided some objectivity and subjectivity, from which the reliability and validity could be identified in terms of quantitative and qualitative data. Including the interviews, the qualitative findings inductively support the quantitative data, providing additional insights from different viewpoint. The formulation and numerical assessment regarding the theory are explained below

#### 4.6.1 Used time

In the first experiment, we collected the time required for the whole session, and determined the average for each quiz. We varied both the time allowed for each question *t* and the number of questions *N* in each quiz. The experiment was separated into 5 different numbers of questions; N=5,10,15,20, or 30. Likewise, given the time allowed, each question was divided into 5 different times: t=5,10,20,30, or 60 s. Time pressure can be considered as the progression of game refinement theory. Typically, the solving rate *v* is defined by using the average amount of time used to answer the questions *AT* and the game length is the total amount of time required to complete whole quiz *T*, with $v_{1}=\frac{AT}{T}$ referring to (18). The game progress model is established from derivation in Section 3.1, which is defined as (19). Thus, we obtained $a_{1}=\frac{2v}{T}=\frac{2\cdot AT}{T^{2}}$ referring to Equation (8).

(18) $$v_{1}=\frac{average\;amount\;of\;answer\;time\;used}{total\;amount\;of\;time\;of\;whole\;quiz}$$

(19) $$a_{1}=\frac{2\cdot average\;amount\;of\;answer\;time\;used}{{\left(total\;amount\;of\;time\;of\;whole\;quiz\right)}^{2}}$$

#### 4.6.2 Quiz scores or answer correctness

Both the second and third experiments focused on the correctness perspective. Varying times allowed for each question *t*, and the numbers of questions *N* were incorporated with differences in difficulties and patterns. The second experiment was separated into three question numbers (N=5,10, or 20) and each question was divided into three different times (t=5,10, or 20 s). The difficulty was categorized into easy, medium, or hard.^2^ The quizzing solving rate was the same as the game progress model's scoring rate by assuming that the quiz score was equal to one correct answer. Therefore, solving rate $v_{1}$ is defined by using the average numbers of correct answers *c* and the total numbers of questions *N* as defined in (20). The objective acceleration $a_{1}$ is defined as (21), where $a_{1}=\frac{2\cdot AT}{T^{2}}$, as defined in (8).

(20) $$v_{1}=\frac{average\;numbers\;of\;correct\;answers}{total\;numbers\;of\;questions}$$

(21) $$a_{1}=\frac{2\cdot average\;numbers\;of\;correct\;answers}{{\left(total\;numbers\;of\;questions\right)}^{2}}$$

Similarly, the third experiment was conducted to examine the impact of various patterns that produced an adjustment of the difficulty level. The third experiment was separated into three question numbers (N=10,20,or 40), and each was allowed one of three different times (t=5,10, or 20 s). The game progress model was the same as in (19) but with a specific difficulty that required technical solving skills.

### 4.7 Qualitative analysis: thematic analysis

The aim of the qualitative analysis was to gain additional insight into the influence of gamification on students' experiences and motivations. Other researchers (Rodrigues et al., 2021) explored a multidimensional approach for personalized gamification considering multiple information sources via thematic analysis to capture and hypothesize users' motivation compared to the traditional implementation of gamification. Others (Dicheva et al., 2015) also conducted a thematic analysis of relevant studies on the use of gamification in the educational context. These studies support our quantitative results and theoretical analysis.

Here, we aimed to understand and explore the impact and perception of participants' subjective experiences a challenge-based gamification activity (Items 1–4). Items 5 and 6 broadened the interview to capture the participants' reactions to and overall motivation regarding challenge-based gamification. In addition, the item's generality (e.g., what do you think) reduced bias, leaving the participant the option to mention specific and additional aspects early in the interview. A previous study described which game elements were examined and implemented, what educational levels were used, and the evaluation outcomes (Dicheva et al., 2015). Unfortunately, no analysis was conducted of the overall impact of gamification on student success in that research.

Instructors play a dominant role in practicing and recognizing gamification, since they act as enablers in the classroom environment. Therefore, a semistructured interview with stakeholders was conducted by Palmquist (2021) which was followed by a thematic analysis. In another study (Bai et al., 2020), the meta-analysis evidence from qualitative studies was integrated using the thematic analysis approach to gain insight into learners' academic performance with gamification intervention.

Thematic analyses were also conducted to extract more personalized information such as participants' experiences, views, and opinions in this study. In another study (Braun and Victoria, 2006), the authors followed the six phases of thematic analysis, where the data were derived from interviews and conversations. Thematic analysis involves identifying the meaning behind patterns through evaluating the themes within the dataset. As thematic analysis tends to be exploratory and driven by the research questions, it can be developed into a coding phase and theme identification.

In this study, the adopted coding was a mixture of inductive and deductive approaches that reflect students' experiences. A data-driven inductive approach defines emergent themes, which assist in deriving meaning and creating themes from data without any preconceptions. The deductive approach formulates the categorization by jumping into the analysis with themes related to the research questions. Typically, this approach is informed by prior knowledge and is uncommon in HCI research (Blandford et al., 2016). This method supports the relationships within the data and provides the flexibility to identify emerging categories from the data. Therefore, semistructured interviews were adopted, which provided a balance between the two approaches and is one of the most commonly adopted qualitative approaches in HCI research (Blandford et al., 2016).

All qualitative data collected were analyzed separately in the data analyzing tool MAXQDA.^3^ All transcripts were reviewed by focusing on exploring conceptual relations and forming patterns (Braun and Victoria, 2006). The clusters and connections of the initial patterns were distinguished during the initial coding. Subsequently, a thematic map was created for clustering the patterns for matching themes, subthemes, and codes. Finally, the results were adopted from methodological and theoretical triangulation, integrating qualitative to quantitative data and interpreting qualitative outcomes through various theoretical perspectives.

## 5 Findings

In this study, we aimed to capture the impact of the variation in challenge-based gamification using the gamified platform as Kahoot! To achieve this, we determined and examined the performance of students using the score rate and used time. These data were calculated by the proposed formulation in order to determine the results and interpretations based on motion in mind. According to Section 3, the motion in mind idea proposes finding motions in an object, allowing such formulation to be described by velocity, force, mass, and energy. This would describe the mechanism of challenge-based gamification in any activity such as those in the education context. Our purpose was to investigate the optimal level of gamification in the activity and state the position of individual motion using both concepts of motion in mind and flow theory to bridge the gap between physics and psychology. A mixed methodology was applied to determine the validity and reliability of this experiment. We first performed a quantitative analysis as a significant part of the study, followed by a qualitative part to gain additional insights. For our quantitative analysis, we conducted three experiments to observe and determine the effects of changes in the parameters based on motion in mind. Velocity *v* and mass *m* are essential indicators used to discover the pattern of challenge-based gamification and other meanings with physics value, including force *F* and potential energy $E_{p}$. Additionally, we interviewed participants to obtain qualitative data, which support the quantitative data in the broader aspects of psychology, such as flow theory and the theory of gamified learning.

### 5.1 Quantitative findings

Since randomization was performed with no control group, we attempted to compare the pre-measurement and post-measurement data, as depicted in Table 5. According to Reeve and Tseng (2011), the typology of engagement in this gamified context was identified and elaborated in a gamification intervention. Two types of engagement were reported as the learning engagement in this study. Consequently, we attempted to investigate occurrences of cognitive and behavior engagement via quiz scores and time used. The results provided preliminary results regarding the setting of N=10 and t=10. A timer can encourage students to focus on the task since the time remaining to complete the task was decreasing. However, the score was inverted so that the students received a higher score for completing the task more quickly This condition resulted in attaining higher learning gains compared to the nongamified condition.

**Table 5:** The pre- and post-test treatment effect of challenge-based gamification experiments.

Pretest	Tot.Ave.	*c*	Post-test	Tot.Ave.	*c*
No-timer	92.5	6.3	Timer	64	7.5
Easy level	60	6.3	Increased level of quiz	76	5.93
Nongamified adaptation	88	3.83	Difficulty randomness	62	7.42
			Sub-goal	72	4.25

Tot. Ave., total average time required; *c*, average number of correct answers.

N=10 and t=10.

Changes in difficulty increased the time required to complete the session and decreased the scores. This increased the difficulty of the challenge-based gamification to higher than the students' skills. This situation reflects that students were cognitively disengaged when the challenge level was too high. The different difficulty levels were used to guide learners in setting achievable goals and developing competencies in a stepwise manner. In this sense, dynamic adaptation could be helpful for further analysis. In the gamified adaptation, the score improved, and the time used decreased. This finding implies that game characteristics influence changes in behavior (Landers, 2014). Specifically, the considered gamified experience significantly encouraged both behavioral and cognitive engagement.

To obtain an in-depth understanding of this gamified experience, we answered the first and second research questions using quantitative analysis. The findings were divided according to the different types of experiments. The analyzed data were computed considering the motion in mind concept.

#### 5.1.1 First experiment: time pressure

Table 6 shows the measures of the game refinement value *GR* and risk chance *m*, based on (18) and (19), respectively. The experiment was conducted three times for several questions where the time used was recorded. Then, the average time for each session and each preference was computed. Determining *GR* involves the time required to answer each question, while question number corresponds to the session's length of time. We observed that the number of questions affected the total time, which explains the decrease in *GR*. This finding implies that time pressure affected the students' engagement (Jaeger and Adair, 2017).

**Table 6:** Measures of game refinement *GR* and risk *m* of Kahoot! with different numbers of questions and question answering times.

Total	Question Time (s)			m=1−v	*GR*
Questions (*N*)	Each	Total	Tot. Ave.		
5	5	25	13	0.480	0.2039
	10	50	23	0.440	0.1356
	20	100	62	0.380	0.1113
	30	150	82	0.450	0.0854
	60	300	191	0.350	0.0651

10	5	50	27	0.460	0.1470
	10	100	64	0.360	0.1131
	20	200	130	0.350	0.0806
	30	300	216	0.280	0.0693
	60	600	495	0.175	0.0524

15	5	75	44	0.413	0.1251
	10	150	102	0.320	0.0952
	20	300	220	0.267	0.0699
	30	450	350	0.220	0.0588
	60	900	850	0.030	0.0458

20	5	100	60	0.400	0.1095
	10	200	116	0.420	0.0761
	20	400	208	0.480	0.0509
	30	600	308	0.490	0.0414
	60	1200	602	0.498	0.0289

30	5	150	105	0.300	0.0966
	10	300	178	0.400	0.0629
	20	600	345	0.425	0.0438
	30	900	488	0.458	0.0347
	60	1800	922	0.487	0.0238

Tot. Ave., total average of time;

m=1−v, risk ratio; GR, game refinement measure.

According to game refinement theory, a sophisticated zone always implies a balance between skill and chance. Most popular games are located in the sophistication zone in the *GR* measure (GR∈[0.07,0.08]), which implies the magnitude of the thrilling sense. Fig. 8 depicts the risk chance of *m* and the *GR* value against the time allowed for each question based on the total number of questions. This gamified platform was achieved with a total question number of 5, 10, or 20, and a time allowed for each question of 20, 10, and 5, respectively. However, when the total number of questions was above 15, the time required for each question was about 7–9 s and less than 5 seconds, respectively. The risk chance *m* tended to increase when N=20 and N=30 because more time was spent answering the question based on the variation in the question time and students' skills. Because of the extra time, it was more likely that the student to doubt their ability to answer the question and would answer it incorrectly.

**Figure 8:** A visualization based on different total question numbers.

Table 7 provides the data analyzed via motion in mind in terms of momentum ($\overset{\to }{p}$) and potential energy ($E_{p}$). The maximum plateau of $\overset{\to }{p}$ was achieved when $m=\frac{1}{2}$, so that $\overset{\to }{p}\leq \frac{1}{4}$. This gamified platform was optimal $\overset{\to }{p}$ when the total question number and time taken for each question were both low (or high) simultaneously. This implies that students could pay more attention in short sessions or long sessions because students were convinced to handle the game, and over time, they identified the competitive aspects. Students might have felt that the intensity was reasonable because of the perceived fairness.

**Table 7:** Measures of momentum $\overset{\to }{p}$, potential energy *E*_*p*_, and risk *m* with different numbers of questions and time allowed to answer the questions.

Total	Question Time (s)		*m*	$\overset{\to }{p}$	*E*_*p*_
Questions (*N*)	Each	Tot. Ave.			
5	5	13	0.480	0.2490	0.2595
	10	23	0.440	0.2484	0.2285
	20	62	0.380	0.2356	0.2921
	30	82	0.450	0.2478	0.2709
	60	191	0.350	0.2313	0.2945

10	5	27	0.460	0.2484	0.2682
	10	64	0.360	0.2304	0.2949
	20	130	0.350	0.2275	0.2957
	30	216	0.280	0.2016	0.2903
	60	495	0.175	0.1443	0.2382

15	5	44	0.413	0.2424	0.2845
	10	102	0.320	0.2176	0.2959
	20	220	0.267	0.1955	0.2868
	30	350	0.220	0.1728	0.2688
	60	850	0.030	0.0524	0.0991

20	5	60	0.400	0.24	0.2880
	10	116	0.420	0.2436	0.2825
	20	208	0.480	0.2496	0.2595
	30	308	0.490	0.2498	0.2564
	60	602	0.498	0.2499	0.2508

30	5	105	0.300	0.21	0.2940
	10	178	0.400	0.2412	0.2863
	20	345	0.425	0.2443	0.2810
	30	488	0.458	0.2482	0.2691
	60	922	0.487	0.2497	0.2559

Tot. Ave.: total average of time;

m=1−v, risk ratio; $\overset{\to }{p}$, momentum; $E_{p}$, potential energy.

$E_{p}$ showed that students obtained motivation from the game. From this result, we found that a total number of questions of 5 or 10 was the best choice to motivate students during this gamified activity. Gamification's positive effect can produce extrinsic motivation in the user in the early stage of the game. Therefore, gamification worked when the total time allowed for the whole session was around 100–150 s. When the risk-taking chance was higher, students may have felt discomfort and lost the desire to continue the game since the game's resistance was greater.

Two parameters are essential to achieve in gamification: acceleration and force. Equation (8) describes the game's acceleration, corresponding to the game refinement measure. The law of conservation of energy is obtained from $E_{p}=\overset{\to }{p_{1}}+\overset{\to }{p_{2}}$, where $\overset{\to }{p_{1}}$ and $\overset{\to }{p_{2}}$ are the objective momentum and subjective momentum, respectively. Subjective acceleration $a_{2}$ is derived from $\overset{\to }{p_{2}}=mv_{2}$, which indicates the subjective aspect of risk-taking chance *m*, and subjective velocity is defined as $v_{2}=2m^{2}-3m+1$. Both measures represent the quantification of player's enforcement in the game; players execute effort to drive the game forward. Objective parameters were considered as the game's ability to build a thrilling experience and create satisfaction.

Table 8 shows that subjective acceleration $a_{2}$ and force $F_{2}$ were negative in every possible setting. Intuitively, a positive force for $F_{1}$ corresponds to players' challenge experienced when playing the game; however, force $F_{2}$ corresponds to a negative acceleration change over risk-taking chance. Games with a small *m* retained negative force $F_{2}$, with a negative peak value at $m=\frac{3}{8}$ where $F_{2}=-0.5625$. This supports the conjecture that low (negative) $F_{2}$ and high (near peak/peak) $E_{p}$ indicate the lowest learning resistance (game's inertia is high) and motivation (high information expectant/availability). The results demonstrate that time pressure can foster engagement and motivation when players are captivated by the game. Notably, a larger *m* seemingly created a greater force, signifying that the intrinsic motivation, even discomfort, dominated this situation.

**Table 8:** Measures of subjective acceleration *a*_2_, subjective force *F*_2_, and risk *m* with different numbers of questions and question times.

Total	Question Time (s)		*m*	$a_{2}$	*F*_2_
Questions (*N*)	Each	Tot. Ave.			
5	5	13	0.480	-1.08	-0.5184
	10	23	0.440	-0.84	-0.4636
	20	62	0.380	-1.48	-0.5624
	30	82	0.450	-1.18	-0.5379
	60	191	0.350	-1.55	-0.5619

10	5	27	0.460	-1.16	-0.5336
	10	64	0.360	-1.56	-0.5616
	20	130	0.350	-1.6	-0.56
	30	216	0.280	-1.88	-0.5264
	60	495	0.175	-2.3	-0.4025

15	5	44	0.413	-1.346	-0.5566
	10	102	0.320	-1.72	-0.5504
	20	220	0.267	-1.93	-0.5155
	30	350	0.220	-2.11	-0.4691
	60	850	0.030	-2.77	-0.1543

20	5	60	0.400	-1.4	-0.56
	10	116	0.420	-1.32	-0.5544
	20	208	0.480	-1.08	-0.5184
	30	308	0.490	-1.05	-0.5126
	60	602	0.498	-1.01	-0.5016

30	5	105	0.300	-1.8	-0.54
	10	178	0.400	-1.37	-0.5585
	20	345	0.425	-1.3	-0.5525
	30	488	0.458	-1.17	-0.5351
	60	922	0.487	-1.05	-0.5116

Tot. Ave.: total average of time;

m=1−v, risk ratio; $a_{2}$, subjective acceleration = 4m−3,

$F_{2}$, subjective force = $ma_{2}$.

#### 5.1.2 Second experiment: difficulty

When applying a challenge that can quickly increase the risk-taking chance, a gamified experience would be obtained if and only if $m\geq \frac{1}{2}$. The various difficulty levels may provoke different aspects of fairness, engagement, and motivation (Denisova and Cairns, 2015; Legaki et al., 2020). This experiment was conducted to observe the effects of alterations in the quiz difficulty to analyze the nature of *m* based on correctness (i.e., how students can obtain information from quizzing). The target quizzes were characterized into three levels; easy, medium, and hard, and distributed in each session. We found that *m* values increased when difficulty was higher since players could not correctly answer the quiz. The difficulty was judged using *m* value in terms of risk frequency ratio, which was used to determined the correctness rate over the total number of questions according to (20) and (21).

Table 9 displays the values of *m*, $\overset{\to }{p_{1}}$, $E_{p}$, and $\overset{\to }{p_{2}}$ for every quiz difficulty level. The results show that most configurations were located in varied risk chance *m*; this formulation reflects the reduction in risk chance *m* based on the total number of questions *N* and time taken *t*. This finding implies that increasing the difficulty of the quiz increased the risk chance; gamified activity was more engaging and risky at the same time. Students become competitive (m>0.5), and devote more effort to the quiz, or stay in the comfort zone (m≤0.5).

**Table 9:** Measures of risk chance *m*, objective momentum *p*_1_, potential energy *E*_*p*_, and subjective momentum *p*_2_ based on variations in the number of questions number and time required for every quiz difficulty level.

*N*	*t*	*T*	difficulty:easy					difficulty:medium					difficulty:hard				
			*c*	*m*	$\overset{\to }{p_{1}}$	$E_{p}$	$\overset{\to }{p_{2}}$	*c*	*m*	$\overset{\to }{p_{1}}$	$E_{p}$	$\overset{\to }{p_{2}}$	*c*	*m*	$\overset{\to }{p_{1}}$	$E_{p}$	$\overset{\to }{p_{2}}$
5	5	25	3.93	0.214	0.1682	0.2644	0.0962	3.3	0.34	0.2244	0.2962	0.0718	2.21	0.558	0.2466	0.218	-0.0286
	10	50	4.66	0.068	0.0634	0.1181	0.0548	3.67	0.266	0.1952	0.2866	0.0914	2.48	0.504	0.2499	0.24798	-0.0019
	20	100	4.83	0.034	0.0328	0.0635	0.0306	4.22	0.156	0.1316	0.2222	0.09058	2.57	0.486	0.2498	0.2568	0.0069

10	5	50	6.9	0.31	0.2139	0.2952	0.0813	5.12	0.488	0.2499	0.2559	0.0059	3.4	0.66	0.2244	0.1526	-0.0718
	10	100	7.5	0.25	0.1875	0.2813	0.0938	5.93	0.407	0.2414	0.286	0.0449	3.93	0.607	0.239	0.188	-0.0511
	20	200	7.93	0.207	0.164	0.2603	0.096	6.1	0.39	0.2379	0.2902	0.0523	4.33	0.567	0.2455	0.2126	-0.0329

20	5	100	8.4	0.58	0.2436	0.2046	-0.0389	6.45	0.678	0.2185	0.1409	-0.0776	5.3	0.735	0.1948	0.1032	-0.0915
	10	200	11.35	0.433	0.245	0.2785	0.0331	6.88	0.656	0.2256	0.1553	-0.0704	5.33	0.734	0.1955	0.1042	-0.0913
	20	400	14	0.3	0.21	0.294	0.084	7.24	0.638	0.231	0.167	-0.0637	5.75	0.7125	0.2048	0.1178	-0.0871

*N*, total questions; c, average numbers of correct answers; m = 1-v, risk ratio;

$E_{p}$ = $\overset{\to }{p_{1}}+\overset{\to }{p_{2}}$; $\overset{\to }{p_{1}}$, objective momentum; $\overset{\to }{p_{2}}$, subjective momentum.

$\overset{\to }{p_{1}}$ indicates the magnitude of engagement in the game, which peaked at pair (N,t)=(20,10) for the easy quiz, (N,t)=(10,5) for the medium difficulty, and (N,t)=(5,10) for the hard quiz. $E_{p}$ describes the potential of a game's movement; peak values were obtained at pair (N,t)=(10,5) in the easy level, (N,t)=(5,5) in the medium level, and (N,t)=(5,20) in the hard level. These results are associated with game engagement when the challenge was introduced, and game curiosity was noted when students felt under control with the appropriate amount of challenge. Highly engaged learners were involved in an arousal situation when m≤0.5, where difficulty reduced curiosity (information expected from learners), while the time and question numbers stabilized with experience to contribute to overall game outcome efficiency.

From another perspective, $a_{2}$ is essential for quantifying $F_{2}$ and for interpreting the context of learning and engagement. Naturally, students solve an easy game with high effort instead of high risk. Adding challenge-based gamification stimulates a student's cognitive curiosity. $a_{1}$ defines the rate of game information over time so that this acceleration will foster a thrill experience for players. As such, players are pushed to play if playing is perceived as accelerating the solving rate. Simultaneously, a large amount of $a_{2}$ can reduce the player's effort based on risk chance. Therefore, a negative value of force $F_{2}$ can be defined as a subjective force that becomes the game's inertial force; in a sense, a negative value is meant to be a force pushing the user to play the game. A negative peak of $F_{2}$ was obtained at $m=\frac{3}{8}$ with $F_{2}=-0.5625$; thus, entry difficulty at various levels affects the change around this negative peak. Hence, time pressure can affect the risk chance, since less time for question answering was associated with higher risk. Therefore, this influenced the student's performance because they had to struggle to complete the task.

$F_{2}$ decreased as players went through the game with less challenge adjustment, and the student anticipated continuing the game. However, $F_{2}$ increased when players went through the game with the added challenge; novice students who did not have many skills felt anxiety corresponding to the amount of challenge adjustment. The least resistance force $F_{2}$ was mostly obtained at the easy and medium levels in this experiment where $m\leq \frac{1}{2}$ (see Table 10). Based on the game progress model, the challenging level seemed to escalate the player's resistance when $m\geq \frac{1}{2}$, denoting a tense situation. This signifies that the game progress model supports the nature of motion in mind, where difficulty adjustment can also push the user to play the game and include more resistance (based on player skill). Thus, player skill would be the main factor required to further visualize the learning context's interpretation.

**Table 10:** Measures of risk chance *m*, subjective acceleration *a*_2_, and subjective force *F*_2_ based on variations in the number of questions and the time for every level of quiz difficulty.

*N*	*t*	*T*	difficulty:easy				difficulty:medium				difficulty:hard			
			*c*	*m*	$a_{2}$	$F_{2}$	*c*	*m*	$a_{2}$	$F_{2}$	*c*	*m*	$a_{2}$	$F_{2}$
5	5	25	3.93	0.214	-2.14	-0.459	3.3	0.34	-1.64	-0.558	2.21	0.558	-0.768	-0.429
	10	50	4.66	0.068	-2.73	-0.186	3.67	0.266	-1.94	-0.515	2.48	0.504	-0.984	-0.496
	20	100	4.83	0.034	-2.86	-0.097	4.22	0.156	-2.38	-0.370	2.57	0.486	-1.056	-0.513

10	5	50	6.9	0.31	-1.76	-0.546	5.12	0.488	-1.05	-0.511	3.4	0.66	-0.36	-0.238
	10	100	7.5	0.25	-2	-0.5	5.93	0.407	-1.37	-0.558	3.93	0.607	-0.572	-0.347
	20	200	7.93	0.207	-2.17	-0.449	6.1	0.39	-1.44	-0.562	4.33	0.567	-0.732	-0.415

20	5	100	8.4	0.58	-0.68	-0.394	6.45	0.678	-0.29	-0.196	5.3	0.735	-0.06	-0.044
	10	200	11.35	0.433	-1.27	-0.549	6.88	0.656	-0.38	-0.247	5.33	0.734	-0.066	-0.048
	20	400	14	0.3	-1.8	-0.54	7.24	0.638	-0.45	-0.286	5.75	0.7125	-0.15	-0.107

*N*, total questions; *c*, average numbers of correct answers; m=1−v, risk ratio;

$a_{2}$, subjective acceleration = 4m−3; $F_{2}$, subjective force = $ma_{2}$.

#### 5.1.3 Third experiment: adaptation of patterns

Usage of randomized difficulty patterns and subgoal patterns provided different learning processes with distinct outcomes in both learning and entertainment (Papp, 2017). Uniform random distribution was applied for the randomized pattern where each question had the same selection chance. This methodology hypothesizes that random distribution improves thrill and creates a challenging experience since it generates uncertainty during the game. This situation describes players leaving their comfort zone but still being conservative as they are encouraged to be in the arousal state; thus, the engagement to keep playing (or learning) is maintained due to players behaving differently. Relative to flow theory (Nakamura and Csikszentmihalyi, 2014), the experimental results show that players developed their skills and started from the anxiety point to the arousal zone, where the optimal condition is to acquire more skills (or information).

Table 11, Table 12 illustrates the experimental results of this adaptation, in which the average number of correct answers *c* is used to describe various motion in mind measures. The *m* for each value was varied, corresponding to each question's time (*t*) and total question number (*N*). The experiment results show the dominant risk ratio where the high uncertainty with a short time allocated for each question was crucial. Additionally, high uncertainty occurred when a higher level of skill was expected in the game. Hence, the sense of engagement and curiosity were uniform based on the motion in mind concept if the appropriate time was established.

**Table 11:** Measures of the physics value of motion in mind and risk *m* for varying numbers of questions and question time with a randomized difficulty distribution.

Total	Question Time (s)		*m*	$\overset{\to }{p_{1}}$	$E_{p}$	$\overset{\to }{p_{2}}$	$a_{2}$	$F_{2}$
Questions (*N*)	Each	c						
10	5	6.33	0.367	0.2323	0.2941	0.0618	-1.532	-0.5622
	10	7.42	0.258	0.1914	0.2841	0.0926	-1.968	-0.5077
	20	7.45	0.255	0.1899	0.2831	0.0931	-1.98	-0.5049

20	5	7.36	0.632	0.2326	0.1712	-0.0614	-0.472	-0.2983
	10	8.27	0.5865	0.2425	0.2005	-0.042	-0.654	-0.3835
	20	8.89	0.5555	0.2469	0.2195	-0.0274	-0.778	-0.4322

40	5	12.3	0.6925	0.2129	0.1310	-0.0819	-0.23	-0.1593
	10	17.85	0.5537	0.2471	0.2205	-0.0265	-0.785	-0.4347
	20	21.33	0.4667	0.2489	0.2654	-0.0165	-1.133	-0.5288

*N*, total questions; c, average numbers of correct answers; m=1−v, risk ratio;

$E_{p}$ = $\overset{\to }{p_{1}}+\overset{\to }{p_{2}}$; $\overset{\to }{p_{1}}=mv$, objective momentum; $\overset{\to }{p_{2}}$, subjective momentum;

$a_{2}$, subjective acceleration = 4m−3;

$F_{2}$, subjective force = $ma_{2}$.

**Table 12:** Measures of the physics value of motion in mind and risk *m* with variations in the number of questions and question time for the subgoal pattern.

Total	Question Time (s)		*m*	$\overset{\to }{p_{1}}$	$E_{p}$	$\overset{\to }{p_{2}}$	$a_{2}$	$F_{2}$
Questions (*N*)	Each	c						
10	5	2.83	0.717	0.2029	0.1148	-0.088	-0.132	-0.0946
	10	4.25	0.575	0.2443	0.2077	-0.0366	-0.7	-0.4025
	20	4.67	0.533	0.2489	0.2325	-0.0164	-0.868	-0.4626

20	5	7.5	0.625	0.2344	0.1758	-0.0586	-0.5	-0.3125
	10	7.83	0.6085	0.2382	0.1865	-0.0517	-0.566	-0.3444
	20	8.23	0.59	0.2419	0.1983	-0.0435	-0.64	-0.3776

40	5	10.45	0.7388	0.193	0.1008	-0.0921	-0.045	-0.0332
	10	11.2	0.72	0.2016	0.1129	-0.0887	-0.12	-0.0864
	20	13.78	0.6555	0.2258	0.1556	-0.0702	-0.378	-0.2478

*N*, total questions; c, average numbers of correct answers; m=1−v, risk ratio;

$E_{p}$ = $\overset{\to }{p_{1}}+\overset{\to }{p_{2}}$; $\overset{\to }{p_{1}}=mv$, objective momentum; $\overset{\to }{p_{2}}$, subjective momentum;

$a_{2}$, subjective acceleration = 4m−3;

$F_{2}$, subjective force = $ma_{2}$.

Intuitively, the negative peak point of $F_{2}$ implies that players were attracted and motivated to continue their activity since this point is recognized as the least resistant to learning. Randomization can create uncertainty and increase the risk ratio (see Table 11). More questions *N* and less time allowed *t* created both feelings of uncertainty and difficulty. Students can acquire skills to deal with such a situation, but they can feel discomfort because of the time pressure. Thus, time pressure and uncertainty influenced students in terms of difficulty, whereas time pressure caused discomfort. When the number of questions ≥20, the risk ratio was too high, and $a_{2}$ converged toward a positive value, implying that students were pushed away from the activity (less attracted by the game).

The subgoal technique was also adopted, which created a clear goal to drive a meaningful activity, including immediate feedback (Nicholson, 2013; Nicholls, 1984). Time, levels, and points were combined in this condition, but the mechanics of this experiment involved forcing the participants correctly answer each question to acquire the right information for the next question. We hypothesized that students would not predict the next question if the current question was regarded as incorrect. Hence, the mechanics might imply a high-risk scenario since students encountered unfamiliar and more complicated tasks. Hence, students would feel contested when time was short with many questions “chaining” (To et al., 2016). This situation is shown in Table 12, where students had an effort at risk ratio of m≥0.5. The feeling of discomfort was high when placing their efforts. The students were aroused and pulled by $a_{2}$, which transitioned them toward performing necessary tasks (high $E_{p}$). This pattern lies in the zone of m≥0.5 where uncertainty and risk are situated, and engagement is expected to be maintained. Most games lie in this zone, indicating that the gamified experience is achieved and low skill is required. Engagement increases as learning growth decreases based on the momentum value of both the objective and subjective factors ($\overset{\to }{p_{1}}$ and $\overset{\to }{p_{2}}$). Adopting this pattern with time pressure and challenge adjustment magnified the uncertainty and lessened the learning potential. However, repetition is the key feature for achieving the ability to recall the information and improve their competence for the next time. The participants with high levels of cognition can be immersed within the activity until they solve the questions. This finding implies this process could possibly be applied in the classroom since it encouraged the students to be engaged during the session. This gamified pedagogy provides an example of activities and quizzes in a practical classroom.

The illustration in Fig. 2(a) outlines the value of solving uncertainty *m* and other physics values when N=10 and t=10. Fig. 9 depicts the value of solving uncertainty *m* regarding the quantity and different kinds of challenge-based gamification. The results show that challenge-based gamification produced changes in the value of *m*. This implies that complexity or uncertainty can increase competitiveness while increasing objectivity. Time pressure, easy difficulty, medium difficulty, and randomization provided m≤0.5, which is more intuition-driven than hard difficulty and subgoal pattern. These results show that time pressure and medium difficulty nearly shifted to the flow zone in which individual ability and activity challenge are equal. This supports the conjecture of gamified learning theory (Landers, 2014; Canhoto and Murphy, 2016) that challenge-based gamification can be used to train and enhance the ability of students while providing challenging tasks. The possible outcome can assist the potential significance and functional relevance of gamification learning and student engagement. The intersection point of subjective force $F_{2}$ and objective momentum $\overset{\to }{p_{1}}$ indicates high-tension excitement, showing the challenge became harder and therefore required more skill. However, the score may rely on the difficulty and complexity that the student faced during different experiences, which affected the difficulty of solving uncertainty *m*. This condition shows that the setting proposed in this experiment can be applied to improve the nongamified condition in the education context.

**Figure 9:** Analogical measure of the physics of all experiments for various masses *m* with *N* = 10 and *t* = 10.

Our application of challenge-based gamification in a gamified platform's context showed an exciting impact. Our findings imply that this technique is essential for changing behavior, which affects improvements in engagement level and learning performance. However, this study's gamified platform was established in a game context and situated in a gamified experience. The game is balanced in terms of skill and chance regarding flow state transition. Thus, it can also be known as gamification, a practical tool that balances “seriousness and fun” and “educational and entertainment” activity as identified previously (Nand et al., 2019). These findings show that gamification should be further developed to provide support in the education domain.

### 5.2 Qualitative findings

Examples of quotes from anonymous interviewees for each code are presented in the coding frame in Table 13. We found justification for applying challenge-based gamification to additionally capture its potential impact from the 10 interviewees. The qualitative results revealed two main themes concerning impacts and perceptions through the intervention of challenge-based gamification in a learning platform. Table 14 displays the counts of the time participants mentioned codes in the interview transcripts and themes.

**Table 13:** Thematic table showing themes, subthemes, and codes obtained from interview transcriptions.

Themes	Subthemes	Codes	Example Quote
Impacts of Challenge-based Gamification	Engagement Impact	Get Aroused	“*I felt aroused, but I had to make an effort.*”
		Competitive	“*I felt competitive, I was encouraged to complete all quizzes.*”
		Anxiety	“*I could not solve the quiz in the first few questions.*”
		Curiosity	“I encountered uncertainty, but this affected my curiosity because of the unknown.”
		Surprised	“Randomization is new to me; I felt surprised in the sense of fun even though I was able to answer correctly.”
		Enjoy	“*The gamified activities were fun and I experienced feelings of curiosity and interest.*”
		Challenging	“*I was very engaged because of time pressure; it was more challenging and required focus.*”
	Learning Impact	Encouragement/Reinforcement	“*The harder level drove my motivation to solve the questions. I could easily answer some of the quizzes and was bored. Then, I would prefer some more challenging tasks so I could learning more than with easier questions.*”
		Development/Learning Improvement	“*I could handle the quizzes better than before, especially with time pressure. I obtained higher and better results in the end.*”
		Concentration	“*I had to pay more attention and focus on the question because of timer.*”
		Creativity	“*After getting used to it, I had to start guessing and considering other options.*”
		Feel Competence/Self-Assessment	“*Gamified quizzing provided me the opportunities to realize the background knowledge.*”

Perceptions of Challenge-Based Gamification	Behavioral Changes	Motivating behaviors	“*It required concentration and motivation to complete the quiz.*”
		Sustaining behaviors	“*Winning was not a target when I tried in this gamified adaptation. I just wanted to go as far as I could depending on my ability.*”
	Intervention efficacy	Allowing learning opportunities	“*When the quiz was not too difficult, I could focus more, which pushed me forward to face the challenge as a new challenge and a new learning opportunity.*”
		Diversity/Variety	“*It was exciting and allowed different students to receive information differently.*”
	Balancing Challenges	Lack of Competence	“*I had little enthusiasm when my abilities were not suited to the quizzing challenges.*”
		Presence of Competence	“*I solved the question that I did not know by myself; I enjoyed meeting the next level of challenges.*”

**Table 14:** Number of mentions by participants of codes relating to this research's themes.

Themes	Number of	Number of participant
	mentions	mentions
	(across all interviews)	(from *n* = 10)
Impacts of Challenge-Based gamification	24	15
Perceptions of Challenge-Based gamification	10	7

#### 5.2.1 Theme 1: Impact of challenge-based gamification

One student declared that they felt excited, but it enabled them to commit extra effort, and this particularly benefited them in terms of increased engagement. One student stated that he perceived competitiveness because he was encouraged to complete all questions in the allotted time. These are considered as excitement and competitiveness, respectively. A little challenge may prompt people in new directions. Surprise and uncertainty with unexpected rewards could keep them engaged and maybe even result in intrinsic engagement in the long term (Carton, 1996). The students' reports showed that uncertainty might increase curiosity since not everything had to be fully explained. Another one stated that “randomization is new to me; it makes me feel surprised but in a fun way because I could answer correctly.” This was also said to impact engagement, both in terms of surprise and curiosity. This statement agrees with that of another student who mentioned that they had more fun and experienced feelings of curiosity and interest. This finding implies that student engagement may be perceived as emotional engagement and subsequently enhanced by curiosity and enjoyment. Most students claimed they perceived that they were more engaged in gamified quizzing and experienced the feeling of being challenged. One mentioned that they felt engaged during time pressure quiz because it was more challenging so they concentrated more than during the quizzes without the extra conditions. This reflects the impact of engagement through encountering challenges.

Engagement retention depends on the individual's skills level regarding difficulty aspects. For instance, in terms of learners, it reflects the confidence that sufficiently improves independent learning. One student stated, “A bit more of a challenge can drive my motivation to answer the questions. I can easily answer some of the quizzes and get bored. Then, I would prefer some challenging tasks to further improve my learning compared to easier questions.” This quote also indicates the impact on learning in terms of encouragement or reinforcement. From a different perspective, further repetition of this experiment could improve their abilities. Some students noted that they could perceive their ability to handle time pressure while improving learning performance through the appropriate use of time and correct answers. This represents the impact on learning in terms of development and improvement. Using the challenge mechanics, students acknowledged that they better gained cognitive skill. For instance, students stated that they had to concentrate on the question since the time was limited. This could be represented as impact on learning in terms of learning concentration. Challenge-based gamification provides the ability to improve their knowledge, and the chance for self-assessment. One student supported this by stating “gamified quizzing provides me the opportunities to realize the background knowledge, and I learned what I did not know, so that made me feel excited.” This represents the impact on learning in terms of competence or self-assessment. There was also positive and negative feelings that indicated resistance in the engagement in this process. A student said, “I could not solve the quiz in the first few questions after I got used to it, so I had to start guessing and considering other options.” This quote can be said to indicate the impact on engagement and learning, both in terms of anxiety and creativity.

#### 5.2.2 Theme 2: Perceptions of challenge-based gamification

Most of the transcription inductively extracted under this subtheme was related to behavior change, intervention efficacy, and balancing challenges. Specifically, we used challenge-based gamification to encourage intended behaviors and sustain behavior change over time. The potential of challenge-based gamification to support the proposed theme was identified through the interviewees' perceptions, including in interview questions, both inductive and deductive. From the last two interview questions, the students reported perceiving the gamified quizzing with challenge-based gamification as positively impacting engagement and learning. Students reported preferring the time pressure mechanics since this produced the sense of achievement when completing the task in a limited time. This implies that students felt motivation, which relates to learning-related behavior. For instance, students were able to learn and improve their abilities through this challenging experience. One of the students claimed, “I could feel pressure when the timer was running. It required concentration and motivation to complete the quiz.” This statement indicates behavior changes in a terms of motivating behaviors. Likewise, challenge-based gamification made students perform autonomously with the motivation to continue and gain in the learning process. One student stated, “Winning was not a target when I tried in this gamified adaptation. I just wanted to go as far as I could depending on my ability.” This statement is also indicative of behavioral changes in a terms of sustaining behaviors.

In terms of intervention efficacy, the students stated that they could engage passively when the quizzes were not too difficult, whereas they had to be proactive during the more difficult quizzes. One of the participants said, “When the quiz was not too hard, I could focus more and was motivated to face each new challenge as a new learning opportunity.” In particular, the challenge and skill relationship mentioned in flow theory could explain the potential of learning opportunities to overcome the current level of performance. This finding can also be represented as allowing learning opportunities. Students experienced diverse sentiments when challenge and uncertainty were added. One mentioned that it was exciting and could allow different students to receive information differently. This finding can also be represented as the efficacy of providing diversity and variety.

Points (correct answers) and levels (difficulty) contributed to users' progression through the system, being the key to identifying where learners could balance the perceived levels of challenge and skill. One asserted that they felt nervous but had a little enthusiasm when their abilities were not sufficient for the quizzing challenges. Another one reported that they were more involved in the learning when their abilities were above the challenge posed by the quizzing. This finding reflects the subtheme of balancing challenges, which could be considered in terms of the lack and presence of competence. One of the main contributions of this study for game design is that there may be an optimal level of perceived time pressure (as a challenge) provided by adjusting mechanics in games that results in maximum competence and performance accompanied by flow and engagement. This relates to the motion in mind concept and flow theory in which optimal control (m<v) and arousal point (m>v) are the boundaries for game design elements. Adaptation may produce the optimal control that suits learning in the long term; here, competence level is above the provided challenge. Time pressure, as a challenge, may produce the optimal arousal that enables engagement in the short term; here, competence level lower than the provided challenge. Creating a challenge in the middle of these two zones might be best for engagement- or learning-related outcomes. The results prove that time pressure can foster engagement and motivation in the zone where players experience arousal and anxiety.

According to the quantitative findings, this mechanic produced a greater force and faster pace. The time element was established by motivating players to pursue desirable goals under pressure. This involved increases in arousal and motor activity. This physical aspect was identified through the interview responses, which were evaluated using keywords, indicating that students entered the arousal zone when they were faced with a shorter allowed time. Another finding linking to the motion in mind concept that this mechanic had nearly the least resistance, which could be taken advantage of to ensure student learning performance through ensuring high curiosity and high expectation within the appropriate time limit.

## 6 Discussion

This study's findings indicate that gamified quizzing positively engages students through entertainment and learning by incorporating challenge-based gamification. The findings suggest that a challenge is an essential element and mechanics in game design, providing a basis for further application in the educational context. The study's findings show that the variation in challenge-based gamification positively contributed to the motion in mind concept, as found from the quantitative study. Since the motion in mind concept also contributed both subjective and objective numerical results, the methodology could be strengthened to incorporate a mixed-methods design to overcome some of the method's limitations. We also conducted a qualitative study to understand the subjective matter more deeply in order to strengthen the concept of motion in mind using from support from flow theory construction.

With mixed success in education, exploring the potential impact of gamification in both the engagement aspect and learning aspects is needed to determine the specific terminologies and processes through which gamification is applied to improve learning. Several approaches were investigated by applying a gamified experience in a learning activity in an ungeneralized scientific way (Landers, 2014; Mitchell et al., 2020). This gap in the knowledge is leading to more studies and discussion on successful gamification. With common ground regarding gamification, some game elements can produce desirable outcomes, which are likely to vary in both the short and long term, depending on the context.

The games should also reflect the skills of the player who learns during the game process. Particularly in a learning environment, an ideal balance between uncertainty and ability is required to emphasize their significance in education and entertainment. Fig. 10 illustrates the allocation of challenge-based gamification related to flow theory; each application is open to interpretation regarding each state of the flow, where risk ratio (*m*) and velocity (*v*) indicate challenge and ability, respectively. This situation explains the impact of *v* and *m* in the transition process of flow where engagement and learning impacts occur.

**Figure 10:** An illustration of challenge-based gamification related to flow theory and motion in mind.

### 6.1 Engagement impact

Maintaining engagement in an activity should be situated on the lowest $F_{2}$ condition, where high $E_{p}$ holds, which indicates the least learning resistance along with high information expectant. Additionally, as observed in quizzing, a situation lacks engagement when the user is uncertain or skills do not progress Engagement can be promoted by having the right level of initial difficulty, so students can progress relative to their ability. If the task is not challenging, the activity might feel monotonous, so the level of difficulty should increased so that the task is entertaining and gives the player a feeling of worthiness and provides effectual meaning.

Here, we found that time limitation promoted the gamified activity's motivation, according to the $\overset{\to }{p_{1}}$ value. As observed in Table 7, Table 8, the $\overset{\to }{p_{1}}$ value was high and gradually decreased during the first phase as the quiz progressed toward the point when the challenge would be adjusted. Additionally, adaptation game mechanics increase user motivation, attenuating the potential impact on engagement caused by uncertainty. When the quizzing involved different challenges with different randomizations each time, the changes ensured the activity remained attractive even though the activity was performed repeatedly. Traditional quiz methods can facilitate engagement by orienting students toward upcoming content and responding to any relevant difficulty. When gamification is adopted, experiencing time pressure may result from the Zeigarnik effect, which focuses people's attention on completing unsolved tasks (Mckinney, 1935) to a certain extent. This implies increases in engagement and curiosity even in students with high cognitive skills.

Kahoot! is a gamified platform that emphasizes time limits for answering and game mastery. Time pressure may be the primary reason the game keeps its players motivated to play. The initial concept was proposed by Jaeger and Adair (2017), who inferred that reducing the amount of time people have to complete tasks motivates them to reflect on the task, and can result in a variety of actions. Based on this evidence, the relationship between the students' engagement level in quizzing is proportional to the potential to acquire information. However, it is crucial to focus on the appropriate level of the challenge, the rate of change of solving uncertainty, and the perceived attraction to ensure the game remains exciting. Thus, an ideal balance between challenge and skill makes the game last longer while positively impacting the player. Therefore, the main aim is to produce a balance between educational value and entertainment, or edutainment, in games. This can be approximated relative to the reasonable zone measures situated at m≤0.5, where learners feel under control when the challenge is adequate. Table 15 summarizes the interpretation of each motion in mind indicator of the three experiments from the engagement perspective.

**Table 15:** An interpretation of each motion in mind indicator for the three experiments from an engagement perspective.

Experiments	Indication	Interpretation
Time pressure	*m* ≤ 0.5 and $\overset{\to }{p_{1}}$	Maintain engagement
	Negative peak *F*_2_ and positive peak *E*_*p*_	Least resistance, high curiosity

Challenge adjustment	balancing *m*	Appropriate difficulty depending on the skills
	Peak $\overset{\to }{p_{1}}$ and *E*_*p*_	Growth rate and stronger motivation

Adaptations of pattern	*m* ≥ 0.5, $\overset{\to }{p_{1}}$ and *E*_*p*_	Hard to maintain engagement
	*a*_2_ and *F*_2_	Negative value arouses students to increase effort

Additionally, we applied a mixed methodology to gain additional insights into challenge-based gamification in an educational setting. We found that students perceived various dimensions of engagement. Considering flow theory, one possible explanation is that every zone can provide students with engagement. However, they may experience competition or anticipation during an activity, which reflects a change in behavior. Supporting this explanation using the physics value, a general effect could be the possible presence of challenge-based gamification that affirms the potential effect proposed by Landers (2014) of the theory gamified learning (game elements influence behavioral changes).

### 6.2 Learning impact

Since gamification does not directly improve learning outcomes, the sense of engagement contributing to the behavior change emerges (Hursen and Bas, 2019). Therefore, learning-related behavior is introduced as an analogical bridge to contribute to the learning outcome (Landers, 2014), emphasizing the development of engagement, which contributes to changing behaviors, where such behaviors generally translate into better learning behavior rather than merely considering the activity outcome. Based on the motion in mind concept, there is still a need to achieve learning-related behavior since each value requires interpretation associated with applying a gamified experience in an education context. The fundamental idea regarding improving learning impact is promoting engagement and the student's emerging potential (i.e., acquiring information). Therefore, students may reveal optimum performance at a moderate challenge level with maximum competence to achieve learning-related outcomes since time pressure creates a challenge. Students' behavior under time limits may be influenced by prior experience, familiarity with the mechanics, and competencies.

Time pressure benefits students by ensuring decision-making is explicitly developed but increasingly harms decision performance and causes suboptimal decisions, which hinder new information or new strategy acquisition (Conte et al., 2015). According to the motion in mind concept, the potential energy value is mostly situated around m=0.33, which implies the least resistance to informational acquisition. Once time pressure is implemented, students tend to encounter risky situations that force students to improve their effort and change their behavior. Other authors (Leroy, 2009) showed that time pressure induces a student to performed an activity more efficiently. However, the amount of information load should be centered on the shortcomings of individual students' memories where learning processing is performed, which is supported by Chang et al. (2018).

The consideration of uncertainty in challenge-based gamification can result in student performance that captures variations in the motion in mind parameters such as $a_{2}$, $F_{2}$, and $E_{p}$. In this study, we found a more balanced distribution of challenge and preferable ability among the students considering the quizzing impact in the classroom, students' skill levels, and students' engagement levels. For a more superficial understanding, the motion in mind *m* value was higher when the gamified platform considered challenge adjustment. Challenge levels must be modified and promoted to improve students' skill levels, as $a_{2}$ and $F_{2}$ are designated as attractiveness and move ability. As described in Table 4, solving hardness (*m*) is regarded as the amount of information students able to retrieve, so that a higher *m* indicates the student was more excited to solve the problem, which improved the learning, as shown in Table 15.

Conversely, a lower *m* value denotes the control state where students can improve their learning without extrinsic motivation (Fig. 10). The impact on student learning was motivated by perceiving information instead, as described by the increases in $a_{2}$ and $F_{2}$. As aforementioned, the negative value of both subjective values means students were pushed towards the activity. Thus, the best conditioning for learning purposes occurs if game elements and well-designed mechanisms are incorporated. We interpret this impact as students feeling a sense of achievement, which reflects learning improvement. The game elements in the current study potentially encouraged students to change their behavior depending on the difficulty of the quiz, as indicated by quiz performance and our quantitative analysis. This supports the qualitative analysis where students provided responses regarding the outcome of the challenge-based design. However, we only applied a quiz with a logical puzzle that was independent of individual skill. As such, we advise caution when interpreting the findings; further studies are required to support these findings.

### 6.3 Practical implications and theoretical contribution

#### 6.3.1 Addressing the conceptual model

This study addressed the research gaps regarding gamification techniques' impacts on learner motivation and engagement. In our study, we discussed student engagement using quantitative findings based on the motion in mind concept outlined by physical values such as velocity, acceleration, momentum, and energy (Iida and Khalid, 2020). Considering this, the study's findings contribute to developing the understanding of this concept by incorporating challenge-based gamification into quizzing, with additional support from qualitative data based on flow analysis.

The findings of this study have two potential practical implications for educational stakeholders: First, the implementation of gamification has benefits in terms of enhancing learning-related behavior. The concept of gamified learning helps the learner and instructor through the learning process, providing engagement and literacy skills. A conceptual scheme was proposed to determine the impacts of gamified learning experience and assessment for the evaluation of learning-related behavior.

Fig. 11 illustrates this study's input–output process of gamification on a gamified platform. The model represents the process of gamification, in which game elements and instructional content are input to drive behavioral changes and engagement. Gamification influences students and their behavior. As such, it often seeks to build upon the increasingly ubiquitous role played by games as an entertainment medium to provide an engaging method to deliver educational content and thus to shift behavior. Our findings and proposed game mechanics can make games particularly appealing as a tool for analyzing and capturing impact by using quizzing. Subsequently, classroom activity can be gamified either for individual users or to comprehensively understand the efficacy of interactive tools. The concepts of challenge-based gamification should be addressed to achieve motivation, which refers to the individual's willingness to remain involved and learning, and the experience of flow. It exhibits the relationship among constructs described in the model and indicates how gamification is intended to influence such outcomes.

**Figure 11:** An input–output process of gamification in a gamified platform.

The application of the gamification process involves considering the design process, including which game elements address the target behavior, and this behavior must have an impact on learning. It specifies that the motion in mind measures the game context related to entertainment and attractiveness, which reflect the engagement aspects. Learning improvement could be encouraged if behavioral changes and motivation occur (Landers, 2014). Thus, both induce learning-related behavior, which affects the capability to improve learning due to gamification. Once motivation is obtained, the result of this improvement is then achievable via effective settings. These experiments provide different gamified learning results and outcomes, but further analysis and designs are needed to support this process.

Similarly, challenge-based gamification can capture its impact on both engagement and learning. With the findings of our studies revealing each game design element's contributions to the challenge experiences, other game elements can be considered and we showed how the these elements can be designed. The mechanics proposed in this study reveal the existence of an optimum time limit, number of questions, and difficulty level through which players experience the flow zone and perform at maximum competence. Moreover, the gamification's features are reflected as mechanic adaptation, which affects students situated in the dynamic zone, which would be useful to promote creative thinking and other meaningful purposes in the education and entertainment contexts. Therefore, stakeholders can benefit from this framework and our approach in this study to create classroom activities to ensure player engagement, achievement, and learning purposes. We provided a promising and innovative method to engage students to learn skills and feel a sense of achievement. This study's findings may help schools transform classroom activities to encourage and retain students' motivation and engagement while challenging and entertaining them.

#### 6.3.2 Impact and perceptions

Participants acknowledged that these interventions are relevant to the motivation and learning process and perceived them as pressing and challenging. The effectiveness of challenge-based gamification is indicated because participants considered the game elements available to them fit their preferences and mentioned that the challenge-based gamification conveyed a sense of flow and curiosity. Also, when using the challenge-based gamification, participants felt the dynamical experience and uncertainty that possibly led to the improvement in the learning process and reinforced the motivation.

Fig. 12 shows the organization of themes, subthemes, and codes, with themes in ovals, subthemes in rounded rectangles, and codes in rectangles. The codes were distributed into five main subthemes, which were distributed into two main themes: (1) impacts of challenge-based gamification and (2) perceptions of challenge-based gamification. Of the five subthemes, two subthemes were clustered under the first theme (impacts of challenge-based gamification): (1) engagement impact and (2) learning engagement. The remaining three subthemes fell under the second theme (perceptions of challenge-based gamification): (1) behavior changes, (2) balancing challenges, and (3) intervention efficacy.

**Figure 12:** Thematic map showing themes, subthemes, and codes.

The mass value *m* denotes the risk chance, with a higher difficulty indicating a lower chance of achieving their desired goals. Here, we found a related basis in flow theory, which specifies a zone of balance between challenge and competence. Levels contain specified elements that create the difficulty. Once the challenge is applied, motivation increases. The motivation level decreases with increasing difficulty, which reflects a high value of *m*. This indicates that difficulty adjustment provides temporal motivation. After the users attempt the harder challenge, they become bored quickly due to the value of force *F*, potential energy $E_{p}$, and momentum $\overset{\to }{p}$. This creates high resistance, resulting in a negative force value, experienced by the student as anxiety and frustration. Therefore, the qualitative findings showed that a sudden increase in challenge level is effective in the short term. To produce long-term results, more than one game element must be incorporated or game mechanics must be adapted.

These results depict the emergence of curiosity, as new pieces of information provide incentives. Cognitive curiosity was exhibited that forced the students to perform flexibly given the uncertainty. According to motion in mind, we proved that quantitative results indicate the relationship between challenge and allocated time. Our qualitative studies proved the conjecture in two ways: First, students enjoyed the process, but engagement was easily lost. Therefore, the appropriate opposing force can take full advantage of the engagement potential. Secondly, opposing forces can result in the decline in learning potential.

Therefore, the results of this qualitative experiment reinforce the theories discussed in this paper. We also found a supplementary result that supports the positive impact of gamification the adoption of game elements, remarkably increasing the dynamics of the elements by adapting the game mechanics with several game elements and finding the optimal prototype of the gamified platform. This ensures with challenging game designs that lead to the use of game elements in the educational classroom.

### 6.4 Limitations and future directions

There are at least two limitations of the current study. First, the challenge-based gamification approach was confined, as mentioned in the methodology section. Therefore, it is difficult to determine which of these components had which effects. The game elements' and our proposed experimental designs would display the different effects of different interpretations. This study may be justified by its internal validity since the proposed design can be used to verify the cause-and-effect relationship established in a study. Nevertheless, external validity could not be achieved since we did not have enough results and the sample size was too small for comparison with other cases. The experimental group was affected because of pre-test measurement, so it would have behaved differently after being exposed to challenge-based approaches.

The challenge-based gamified experience is also limited to motivating students in a high-risk situation and effectively producing a more engaging activity. Hence, as engagement and motivation increase, the interpretation of learning via quizzing may be flawed, thus making it challenging to analyze the approach further and rationalize the conceptual scheme (Fig. 11). As such, this limitation suggests caution when interpreting the results since such findings were not externally validated, requiring further investigation. Future studies should also consider complex details when designing engaging gamified activities and experiments in educational settings.

Secondly, we aimed to bridge the gap between motion in mind and flow theory. The proposed interpretation might work in the current circumstances, but it may not work for different mechanisms (i.e., other gamification approaches). Our findings may require an extension of underlying psychological analysis or dynamic mechanisms to provide insights into entertainment and learning experience through gamification to highlight this limitation. A future study could investigate the use of a dynamic approach: a more objective method that can be seen explicitly, or a complex methodology, including specific artificial intelligence coping with different participants. Furthermore, two alternative methods to improve student skill and contribute a dynamic approach: growth rate as described by Agarwal et al. (2019) and dynamic adjustment as described Sepulveda et al. (2019), could be used to visualize and clarify the current contextual gap existing in learning to bridge the gap between flow theory and motion in mind.

## 7 Conclusions

Gamification has become a promising direction in nongame alignments. The gamification approach involves a process used across various contexts to engage and develop a particular behavior (Deterding et al., 2011). Behaviors are the proximal impacts that should be assessed unless the impact of gamification and transition behaviors were misunderstood. Challenge-based gamification provides a precise approach that examines which element contributed to learning and induces a specific outcome.

From this study, we conclude that gamification effort empirically increases engagement and emergence behaviors. Here, we used challenge-based gamification in a quizzing activity to encourage student motivation based on motion in mind interpretation. First, we examined the impacts of time pressure and difficulty on the feelings of curiosity and uncertainty. Both ultimately affected the engagement- and learning-related outcomes of applying quizzing and educational content into a gamified platform. The motion in mind concept proposed here provides measurements of engagement, motivation, and the nature of the mind in various contexts and from various perspectives. This approach identifies two specific methods through which gamification can moderate experiences and affect a learning-related behavior.

Our findings also showed that gamified quizzing improves classroom activity by referring to flow theory since the challenge shifts students' experience into an arousal zone, which subsequently transforms if the challenge and students' abilities are encouraged, which can be achieved using the gamified elements proposed in this paper. This shows that the learning performance improved, as represented by the learners' performance metrics, leading to learning impact being situated in the control zone. Thus, we strongly recommend that further studies be conducted in order to implement such dynamic gamified quizzes with other gamification designs and elements to support the understanding and the transition of engagement- and learning-related behavior in the education context.

## Declarations

### Author contribution statement

Punyawee Anunpattana: Conceived and designed the experiments; Performed the experiments; Analyzed and interpreted the data; Contributed reagents, materials, analysis tools or data; Wrote the paper.

Mohd Nor Akmal Khalid and Hiroyuki Iida: Conceived and designed the experiments; Analyzed and interpreted the data; Contributed reagents, materials, analysis tools or data; Wrote the paper.

Wilawan Inchaman: Analyzed and interpreted the data; Contributed reagents, materials, analysis tools or data.

### Funding statement

This work was supported by 10.13039/501100001691Japan Society for the Promotion of Science (19K22893).

### Data availability statement

Data will be made available on request.

### Declaration of interests statement

The authors declare no conflict of interest.

### Additional information

Supplementary content related to this article has been published online at https://doi.org/10.1016/j.heliyon.2021.e08637.

No additional information is available for this paper.

## Appendix A Interview questions

1. What do you think are the significant impacts of the three different challenge-based approaches on gamified quizzing?
  (a) How was your motivation/engagement?
  (b) How was your learning achievement?
2. What did you feel about your involvement during the time pressure gamified experience?
3. What did you feel about your involvement with the variation in the quizzes' difficulty?
4. What did you feel about your involvement during the adaptation of quizzing (subgoal and random difficulty)?
5. Which kind of gamified quizzing did you prefer?
6. What benefits did you obtain from challenge-based gamification?

## Appendix B Supplementary material

mmc1.docx Appendix A - Interview Questions. mmc1.docx

## Footnotes

1 https://kahoot.com/.

2 https://hitbullseye.com/puzzle/easy-logic-puzzles.php.

3 https://www.maxqda.com/.
